# Facial Recognition System Based on Genetic Algorithm Improved ROI-KNN Convolutional Neural Network

**DOI:** 10.1155/2022/7976856

**Published:** 2022-10-10

**Authors:** Xiao Wang, Yan Li

**Affiliations:** Xi'an FanYi University, Xi'an, 710105 Shaanxi, China

## Abstract

The facial recognition system is an application tool that uses artificial intelligence technology and biometrics technology to analyze and recognize the facial feature information of the human face. It is widely used in various fields, such as attendance and access control management in schools and companies, identity monitoring in stations and stores, facial recognition for fugitive criminals, and facial payment on mobile terminals. However, due to the short development time of the facial recognition system, the facial recognition system has the problem of low recognition accuracy when the recognized object is not cooperative. Although some scholars have proposed the region of interest (ROI)-K nearest neighbor algorithm (KNN) convolutional neural network theory by using the ROI and KNN and applied it to face recognition, the facial recognition system based on ROI-KNN convolutional neural network did not solve the problems of insufficient facial recognition accuracy and insufficient security. Under the conditions of insufficient illumination, excessive expression change, occlusion, high similarity of different individuals, and dynamic recognition, the recognition effect of the facial recognition system based on the ROI-KNN convolutional neural network is relatively limited. Therefore, to make the recognition accuracy of the facial recognition system higher and to make the facial recognition system play a greater role in the social and economic fields, this paper used the adaptive quantum genetic algorithm, the improved marker line graph genetic algorithm, and the feature weight value genetic algorithm to study the facial recognition system of the ROI-KNN convolutional neural network. The research results showed that after improving the ROI-KNN convolutional neural network based on the genetic algorithm, the recognition accuracy of the facial recognition system was increased by 4.99%, the recognition speed was increased by 7.46%, and the recognition security was increased by 2.66%.

## 1. Introduction

With the development of artificial intelligence technology and biometric technology, facial recognition systems are widely used in social and economic fields. As an emerging thing, the facial recognition system has not been developed for a long time. Although some scholars have established a facial recognition system based on the region of interest-K nearest neighbor algorithm (ROI-KNN) convolutional neural network, the accuracy and security issues of facial recognition are still not solved. Therefore, the use of the genetic algorithm in this paper to improve the ROI-KNN convolutional neural network facial recognition system has practical value and is necessary.

The rapid development of artificial intelligence technology has provided a good development environment for facial recognition systems, and many scholars have conducted research on facial recognition systems. Majumder et al. proposed a novel automatic facial expression recognition system using a deep network framework to make facial recognition networks more computationally efficient and more accurate in terms of performance [1]. Siddiqi trained facial recognition expressions through Hidden Markov Models and used new feature extraction methods to improve the cognitive accuracy of facial recognition systems. The research results were utilized to propose a real-time facial expression recognition (FER) system for facial recognition systems [2]. Banerjee et al. proposed a crow search algorithm based on the Brownian motion adaptive neuro-fuzzy inference system and proposed four steps for face recognition using the facial recognition system in detail [3]. Saxena et al. studied and analyzed the integrated network and emotion recognition of facial recognition systems, and established a valence model for facial recognition and emotion classification [4]. Karthick et al. believed that traditional manual attendance not only takes time and energy but also has low efficiency and high error rate, and established a facial recognition attendance system through research on facial recognition [5]. He considered the influence of glass on facial recognition in the process of researching facial recognition systems and believed that further testing and analysis should be carried out on the face images collected from glass [6]. Cheng et al. proposed to use two-layer convolutional neural network learning to sparsely represent the high-level features of face recognition and established a sparse representation classifier system for face recognition [7]. Although scholars have done a lot of research on facial recognition systems, the research on facial recognition systems based on ROI-KNN convolutional neural networks was relatively small. Therefore, this paper studied the facial recognition systems based on ROI-KNN convolutional neural networks.

The ROI-KNN convolutional neural network combined the region of interest and the KNN. As one of the representative algorithms of deep learning, it is often applied to research in various fields. Jian et al. studied the identification and classification of fingerprints and proposed a new fingerprint classification algorithm using the ROI-KNN convolutional neural network, which improved the accuracy and speed of fingerprint identification [8]. Yin et al. believed that the short-text classification algorithm had the problem of data sparse, and based on the ROI-KNN convolutional neural network, a neural network language model for short text was proposed [9]. Kim et al. used convolutional neural networks to study the characteristics of unsupervised learning and came to the conclusion that unsupervised learning had advantages over supervised learning [10]. Iglovikov et al. applied a convolutional neural network to multispectral data processing and proposed a detection method for satellite image features [11]. Yuan et al. proposed a two-stream parallel interactive convolutional neural network through research on the application of convolutional neural network, which has played a significant role in the disease identification of crop leaves [12]. Sheng and Zhao used the convolutional neural network and KNN algorithm to research and analyze handwriting recognition and established a digital recognition model, which further improved the accuracy of handwriting recognition [13]. Shen made a comparative evaluation of the application in the field of facial emotion classification using the ROI-KNN convolutional neural network and proposed a new deep learning training improvement scheme for facial expression classification [14]. Although the above scholars have conducted research on convolutional neural networks and ROI-KNN convolutional neural networks, with the development of science and technology, facial recognition equipment with more complex functions and higher recognition accuracy requirements also appears, and the technicality of ROI-KNN convolutional neural network faces the common challenges of facial recognition equipment and the recognition environment. Therefore, this paper studied the improvement of ROI-KNN convolutional neural network based on a genetic algorithm, so as to make the facial recognition system based on the ROI-KNN convolutional neural network more efficient.

To make the ROI-KNN convolutional neural network further exert its advantages in the field of facial recognition and improve the recognition accuracy and recognition speed of the facial recognition system, the improved face recognition system based on the ROI-KNN convolutional neural network was studied by using adaptive quantum genetic algorithm, improved marker line genetic algorithm, and feature weight value genetic algorithm in this paper.

## 2. Evaluation of the Improvement of ROI-KNN Convolutional Neural Network Based on Genetic Algorithm

### 2.1. Basic Convolution Block under ROI-KNN Convolutional Neural Network Structure

Compared with the basic convolution block of the ROI-KNN convolutional neural network, the basic convolution block of the ROI-KNN convolutional neural network improved based on the genetic algorithm, which is more complex in structure, as shown in Figure 1.

As can be seen in Figure 1, after the improvement of the genetic algorithm, there are 4 parallel lines in the basic convolution block under the ROI-KNN convolutional neural network structure. When obtaining information in different spaces, to reduce the amount of data calculated by the model, the two middle lines will first perform 1 × 1 convolution on the input. Appropriate padding is used for all 4 lines to make the height and width of the input and output consistent, which also makes the structure and lines of the basic convolution block more reasonable.

### 2.2. Architecture of ROI-KNN Convolutional Neural Network

The ROI-KNN convolutional neural network is widely used in the field of image recognition [15]. In this paper, after researching the ROI-KNN convolutional neural network using the genetic algorithm, the architecture of the ROI-KNN convolutional neural network is established, and the specific content is shown in Figure 2.

As can be seen in Figure 2, the architecture of the ROI-KNN convolutional neural network established in this paper based on the genetic algorithm is divided into four parts: input layer, convolution layer, pooling layer, and connection layer. In the ROI-KNN convolutional neural network, the input layer usually represents an image with a pixel matrix. Starting from the input layer, the ROI-KNN convolutional neural network can convert the image 3D matrix of the previous layer to the next layer through different network structures. The convolutional layer is the most critical part of the convolutional neural network. In the ROI-KNN convolutional neural network, the operation of the pooling layer is similar to converting a high-pixel image into a low-pixel image. The purpose is to reduce the number of nodes in the connection layer and the parameters in the convoluted neural network. After several rounds of processing of convolutional layers and pooling layers, image information will be converted into feature information suitable for convolutional neural networks, and then the connection layer can be used to complete the classification task.

### 2.3. Application of ROI-KNN Convolutional Neural Network Facial Recognition System

The rapid development of artificial intelligence technology and biometric technology has made facial recognition systems widely used in people's production and life, such as face recognition attendance access control systems, identity recognition monitoring systems in shopping malls and stations, etc. [16]. The content is shown in Figure 3.

As can be seen in Figure 3, the improved ROI-KNN convolutional neural network facial recognition system can be applied to attendance and identity recognition. Servers, switches, and communication networks ensure the normal operation of the facial recognition integrated machine. The facial recognition integrated machine is used as the acquisition subsystem of facial recognition, which is responsible for capturing the information of facial features. After the facial recognition integrated machine completes image acquisition and face positioning, the subsystem is responsible for the transmission of image information and back-end analysis. The improved facial recognition system usually uses data compression technology in information transmission to save storage space and improve transmission efficiency. Back-end analysis is to analyze the information features of the face and compare it with the facial features of the database to determine whether someone's facial feature information matches the facial feature information recorded in the database at this time.

## 3. Improvement of the Utilization Algorithm of ROI-KNN Convolutional Neural Network

### 3.1. Adaptive Quantum Genetic Algorithm

The genetic algorithm is an algorithm that uses computer technology and mathematical thinking to simulate the natural evolution process and converts the solving process of problems in other fields into the process of chromosome crossover and mutation in the biological field [17]. Based on the genetic algorithm, this paper proposes an adaptive quantum genetic algorithm with a better effect on improving the ROI-KNN convolutional neural network.

Assuming the initial chromosome is {*M*_1_(*s*) *M*_2_(*s*) *M*_*N*_*m*__(*s*)}, there are:

(1) $$\begin{array}{c} M_{p}\left(s\right)=\left\{\begin{array}{c} y_{p1}^{s}\;y_{p2}^{s}\;y_{{pN}_{h}}^{s}\\ \lambda_{p1}^{s}\;\lambda_{p2}^{s}\;\lambda_{{pN}_{h}}^{s} \end{array}\right\}\left(p=1,2,...,N_{m}\right). \end{array}$$

Among them, *y*_*pq*_^*s*^ represents the real encoded value and *λ*_*pq*_^*s*^ represents the qubit phase angle.

The formula for calculating the probability amplitude is:

(2) $$\begin{array}{c} \left[\begin{array}{c} \mu_{pqc}^{s}\\ \nu_{pqc}^{s} \end{array}\right]=\left[\begin{array}{c} \cos\theta \;\sin\theta \\ -\sin\theta \;\cos\theta \end{array}\right]\left[\begin{array}{c} \mu_{pqc}^{s-1}\\ \nu_{pqc}^{s-1} \end{array}\right]. \end{array}$$

The formula for calculating individual elements is:

(3) $$\begin{array}{c} M_{pqc}^{s}={\left(\mu_{pqc}^{s}\right)}^{2}\left(M_{c\max}-M_{c\min}\right)+M_{c\min}. \end{array}$$

Among them, *α*_*pqc*_ is the *c* element of *Z*_*pq*_, *λ*_*pqc*_^*s*^ = *λ*_*pqc*_^*s*−1^ + *α*_*pqc*_*θ*^″^ and *θ* are the changes of the angle, and *λ*_*pqc*_^*s*^ is the rotation angle.

The optimal individual represents the allowable range of individual elements, there are:

(4) $$\begin{array}{c} M_{c\max}=\max\left(M_{\text{best}c},D_{p}^{s}\right), \end{array}$$

(5) $$\begin{array}{c} M_{c\min}=\min\left(M_{\text{best}c},D_{p}^{s}\right). \end{array}$$

The calculation method of individual elements is called way 1, and the way of expressing the allowable range of individual elements by the optimal individual is called way 2. Their use frequency ratio formula is:

(6) $$\begin{array}{c} \left\{\begin{array}{c} E_{\text{way}1}=\left(90-\frac{80s}{S}\right)/100\\ E_{\text{way}2}=\left(10+\frac{80s}{S}\right)/100 \end{array}\right., \end{array}$$

where *E*_way1_ and *E*_way2_ are the usage frequency ratios of way 1 and way 2, respectively, *s* is the current evolutionary algebra, and *S* is the total evolutionary algebra for each calculation cycle.

### 3.2. Improved Marker Line Graph Genetic Algorithm

The genetic algorithm for labeling line graphs is a method that applies genetic algorithms to the field of line graph labeling and uses genes and chromosomes to represent line graphs for research [18]. In this paper, the method of adaptive parameter adjustment is adopted, and the genetic algorithm of the marker line graph is studied so that the improved marker line graph genetic algorithm can play a better effect in the process of improving the ROI-KNN convolutional neural network.

The global probability of the line graph is:

(7) $$\begin{array}{c} I\left(H\right)=\frac{\overset{S}{\underset{s=1}{\sum }}I\left(H_{s}\right)}{S}. \end{array}$$

The node probability expression derived from the Bayesian model is:

(8) $$\begin{array}{c} I\left(H_{s}\right)=\frac{{\left(1-i\right)}^{S}}{\left|\alpha_{s}\right|}\underset{h\in \alpha_{s}}{\sum }{\left[\frac{i}{1-i}\right]}^{L_{s,h}}. \end{array}$$

Among them, *L*_*s*,*h*_ represents the distance between the current mark of the node and the corresponding node element *h*.

Assuming *p* is the error-free probability of the labeling process, formula (8) can be rewritten as:

(9) $$\begin{array}{c} I\left(H_{s}\right)=\frac{{\left(1-i\right)}^{S}}{\left|\alpha_{s}\right|}\underset{h\in \alpha_{s}}{\sum }\exp\left[-L_{s,h}\;\ln\frac{1-i}{i}\right]. \end{array}$$

The minimized value function formula of the line graph marker obtained from formula (9) is:

(10) $$\begin{array}{c} D\left(H\right)=\overset{S}{\underset{s=1}{\sum }}\underset{h\in \alpha_{s}}{\min L_{s,h}}. \end{array}$$

The fitness function of the chromosome is:

(11) $$\begin{array}{c} E\left(m\right)=\exp\left[-{wD}_{m}\left(H\right)\right]. \end{array}$$

Among them, w is an introduced scaling parameter related to the number of algorithm iterations.

The expression for the scaling parameter is:

(12) $$\begin{array}{c} W=\frac{q^{1/l}}{D_{\max}\left(H\right)}, \end{array}$$

(13) $$\begin{array}{c} l=1+\mathrm{lg}\left(S\right). \end{array}$$

Among them, *D*_max_(*H*) is the maximum value of the chromosome value function, *S* is the maximum number of iterations, and *q* is the current number of iterations.

Assuming that the current fitness of the calculated chromosome is *E*_(*m*)_, the probability of individual m being selected is:

(14) $$\begin{array}{c} F\left(m\right)=\frac{{\left[E\left(m\right)\right]}^{2}}{\overset{i}{\underset{m=1}{\sum }}{\left[E\left(m\right)\right]}^{2}}. \end{array}$$

The cumulative probability of individual m being selected is:

(15) $$\begin{array}{c} G_{m}=\overset{m}{\underset{l=1}{\sum }}F\left(l\right). \end{array}$$

Among them, in *F*(*m*), a value *v* between 0 and 1 is selected. When *v* ∈ (*G*_*m*=1_, *D*_*m*_), the *m* individual is selected. The above operation is repeated *i* − 1 times until *i* − 1 chromosomes are selected.

### 3.3. Genetic Algorithm for Feature Weight Values

The feature weight value genetic algorithm is a method that uses the genetic algorithm to extract and optimize the image features to obtain the optimal solution of the feature weight value [19]. In this paper, the feature weight value genetic algorithm is applied to the improvement of the ROI-KNN convolutional neural network to improve the effect of image classification and face recognition.

Image color and texture features are extracted and combined to get the final vector:

(16) $$\begin{array}{c} T\left(J,I\right)=\overset{k}{\underset{p=1}{\sum }}v_{p}\sqrt{{\left(f_{Jp}-f_{Ip}\right)}^{2}}. \end{array}$$

Among them, *J* is the example image, *I* is the target image, *k* is the number of features, and *v*_*p*_ is the weight.

The optimal weights for image classification and face recognition are:

(17) $$\begin{array}{c} G=f\left(V\right)=\overset{K}{\underset{p=1}{\sum }}\sqrt{AT}. \end{array}$$

Among them, *K* is the number of images, and $\sqrt{AT}$ is the precision and precision.

The convolutional neural network is optimized by the genetic algorithm of feature weight value, and the weight update formula is:

(18) $$\begin{array}{c} V^{\left(s\right)}=V^{\left(s-1\right)}-\beta \frac{\kappa Q\left(v,c,\lambda \right)}{\kappa V}\left|{}_{V=V^{\left(s-1\right)}}\right., \end{array}$$

(19) $$\begin{array}{c} c^{\left(s\right)}=c^{\left(s-1\right)}-\beta \frac{\kappa Q\left(v,c,\lambda \right)}{\kappa c}\left|{}_{c=c^{\left(s-1\right)}}\right., \end{array}$$

(20) $$\begin{array}{c} \lambda^{\left(s\right)}=\lambda^{\left(s-1\right)}-\beta \frac{\kappa Q\left(v,c,\lambda \right)}{\kappa \lambda }\left|{}_{\lambda =\lambda^{\left(s-1\right)}}\right.. \end{array}$$

Among them, *V* is the weight of the optimized convolutional neural network, *c* is the bias value, *λ* is the weight parameter, and *s* represents the current layer in the convolutional neural network.

## 4. Experimental Design of Facial Recognition System Evaluation

In this paper, 50 experimental personnel in a certain area were selected according to factors such as age and gender, and they were divided into two groups under the condition that the age and gender of the two groups were not significantly different. There were 25 people in each group, and each group contained 5 pairs of people with high facial similarity. A group using the improved ROI-KNN convolutional neural network facial recognition system based on the genetic algorithm was tested, called the experimental group, and called this facial recognition system as the improved ROI-KNN facial recognition system. Another group was tested with a facial recognition system based on the ROI-KNN convolutional neural network, called the control group, and called this facial recognition system as the ROI-KNN facial recognition system. The facial recognition system was used to conduct 100 face recognition tests on each person in different environments, and the data were stored and organized for experimental analysis.

## 5. Experimental Results and Evaluation of Facial Recognition System

### 5.1. Facial Recognition Accuracy

#### 5.1.1. Facial Recognition in Low-Light Environments

Lighting change is one of the key factors affecting face recognition. Faces have three-dimensional structural features. The intensity of light and the shadows cast will obviously affect the original facial features. Insufficient light will lead to a decrease in the recognition accuracy of the face recognition system, which will reduce the practicability of the face recognition system. The specific face recognition data in an environment with insufficient light is shown in Figure 4.

It can be seen in Figure 4 that the overall recognition accuracy of the experimental group is greater than that of the control group, which shows that the recognition accuracy of the facial recognition system is significantly improved after using the genetic algorithm to improve the ROI-KNN convolutional neural network. From the data of the third to seventh experimenters, the recognition accuracy of the ROI-KNN facial recognition system exceeds that of the improved ROI-KNN facial recognition system. It may be due to the specialization of sample individuals or the way individuals are arranged and combined that affect the experimental data, but it does not affect the scientificity and rationality of the experimental results. From an individual point of view, the improved ROI-KNN facial recognition system has a maximum facial recognition accuracy rate of 98% in a low-light environment, while the ROI-KNN facial recognition system has a maximum of 90%, a difference of 8%. It shows that the improved ROI-KNN facial recognition system can still play a better role in a low-light environment and has good recognition and adaptability. Compared with the control group, the average recognition accuracy rate of the experimental group increases by 5.71%, indicating that the improved ROI-KNN facial recognition system can play more roles in the environment of insufficient lighting and has more practical values.

#### 5.1.2. Facial Recognition under Different Expression Changes

In addition to considering lighting conditions, facial recognition systems also need to consider the impact of facial expression changes on face recognition. Emotions such as crying, laughing, and anger will greatly change facial features, which greatly affects the judgment of the facial recognition system. The specific research content is shown in Figure 5.

As can be seen in Figure 5, in the experiment of this paper, the three expression changes of crying, laughing, and anger have the greatest impact on facial recognition, crying, followed by laughing, and the emotion that has the least impact on facial recognition is anger. The emotion caused by crying changes greatly, so whether it is the ROI-KNN facial recognition system or the improved ROI-KNN facial recognition system, the facial recognition accuracy under the expression of crying is low. However, compared with the ROI-KNN facial recognition system, the recognition accuracy of the improved ROI-KNN facial recognition system is 4% higher in crying emotions, and the improved ROI-KNN facial recognition system is still effective. The average recognition accuracy of the improved ROI-KNN facial recognition system under the three expressions of crying, laughing, and anger is 76.67%, while the ROI-KNN facial recognition system is 71.67%. Compared with the ROI-KNN facial recognition system, the average recognition accuracy of the improved ROI-KNN facial recognition system is increased by 5%. In the case of different expression changes, the improved ROI-KNN facial recognition system has more advantages.

#### 5.1.3. Facial Recognition under Occlusion

In real life, the objects recognized by the face recognition system are not all complete facial features. For example, people will wear sun hats for sun protection and masks for public health reasons. Sun hats and masks will affect the recognition accuracy of the facial recognition system. The specific facial recognition data in the occluded state are shown in Figure 6.

As can be seen in Figure 6, there are not many experimenters with a recognition accuracy rate of 80%. It seems that masks and sun hats have a great impact on facial recognition. In the experimental group, there are 7 people with a recognition accuracy rate of 80%, while there is only one person in the control group. It shows that the improved ROI-KNN facial recognition system can still maintain a relatively good recognition accuracy under the occlusion state. The recognition accuracy of the improved ROI-KNN facial recognition system is not high at the beginning, only 63% at the beginning. However, as the test continues, the recognition accuracy data are on the rise in a fluctuating state, indicating that the improved ROI-KNN facial recognition system has a strong learning ability, and the more recognition times, the stronger the ability to recognize images and faces. The average recognition accuracy of the experimental group is 75.16%, and that of the control group is 72.64%, which is an increase of 2.52%, indicating that the improved ROI-KNN facial recognition system has more advantages in the occlusion state.

#### 5.1.4. Facial Recognition under the Condition of High Degree of Face Similarity

On the whole, since the structure and shape of the face structure are very similar, the difference between different individuals is not very large. From an individual point of view, due to genetic and environmental factors, there will be two extremely similar individuals in a certain area, not to mention the degree of facial similarity of identical twins. The specific research contents under the condition of a high degree of face similarity are shown in Table 1 and Figure 7.

It can be seen from Table 1 and Figure 7 that although the similarity of each pair of experimenters in the two groups is close, the experimental results of the two groups are also different. From the overall data, the recognition accuracy of the experimental group is gradually increasing, and the recognition accuracy has increased from 69% to 81%. It can be seen that the improved ROI-KNN facial recognition system has strong adaptability to the recognition environment. The experimental data of the control group are high and low, and the ROI-KNN facial recognition system is not stable in identifying two similar individuals. The average recognition accuracy of the experimental group is 76.8% and that of the control group is 71%. The average recognition accuracy of the experimental group is 5.8% higher than that of the control group.

#### 5.1.5. Facial Recognition under Dynamic Recognition Conditions

In the practical application of facial recognition systems, facial recognition is not always carried out in a static environment, such as facial recognition in subways, supermarkets, and face detection at station checkpoints. Facial recognition under dynamic recognition conditions will result in blurred facial images or inaccurate focus of the camera, which will affect the recognition accuracy of the facial recognition system. The specific data content is shown in Figure 8.

As can be seen in Figure 8, the facial recognition accuracy data of the experimental group and the control group are generally not very high. In a dynamic environment, due to the camera quality, network transmission volume, system computing power, and other issues, coupled with the low resolution of the collected facial images, the accuracy of facial recognition is lower than that in a static environment. Judging from the high recognition accuracy of individuals, there are 5 experimenters in the experimental group whose recognition accuracy reaches 80%, while those in the control group do not reach 80%. It can be seen that under the condition of dynamic recognition, the improved ROI-KNN facial recognition system has more development potential. From the average recognition accuracy rate, the average recognition accuracy rate of the experimental group is 69.72%, and the average recognition accuracy rate of the control group is 63.8%. The improved ROI-KNN facial recognition system improves dynamic recognition by 5.92% compared with the ROI-KNN facial recognition system.

### 5.2. Facial Recognition Speed

In addition to the recognition accuracy, the speed of facial recognition is also an important factor affecting the effect of facial recognition. In this paper, the average recognition speed is calculated based on the recognition speed of the two groups of people in 5 different recognition environments. The specific content is shown in Figure 9.

As can be seen in Figure 9, regardless of whether the experimental group or the control group, the facial recognition speed has reached within 1 second, and the method of observing and recording with the naked eye can no longer meet the needs of this experiment. Therefore, this paper loads an automatic timing program in the facial recognition system to help the experiment go on smoothly. On the whole, although the recognition time data of the experimental group is higher in the first few times, as the test progressed, the overall recognition time spent on the whole is developing in a downward trend. The average facial recognition time spent in the experimental group is 0.645 seconds, and the control group is 0.697 seconds, a difference of 0.052 seconds. This equates to an average facial recognition speed of 7.46% for the experimental group compared to the control group.

### 5.3. Facial Recognition Security

In addition to the recognition accuracy and recognition speed, the facial recognition system also needs to consider recognition security issues. In this paper, the security of the facial recognition system is studied by simulating a real face with two-dimensional photographs, simulating a face structure with a 3D model, and testing a network image grafting recognition. The specific content is shown in Figure 10.

As can be seen in Figure 10, in the security test of two-dimensional images, the ROI-KNN facial recognition system and the improved ROI-KNN facial recognition system performed relatively well. With the development of artificial intelligence technology and biometric identification technology, researchers have matured in the research on the informatization characteristics of human face structure, and traditional two-dimensional images have been difficult to deceive new face recognition systems. However, the security index of the ROI-KNN facial recognition system was not 100%, indicating that the improved ROI-KNN facial recognition system was more stable and secure in the recognition process. The average safety index of the experimental group was 98.33%, and the average safety index of the control group was 95.67%. Compared with the control group, the average security index of the experimental group increased by 2.66%, indicating that the improved ROI-KNN facial recognition system has a more obvious role in solving the security problem of facial recognition and has a broader development prospect.

## 6. Conclusion

Although the facial recognition system was widely used in the social and economic fields, the facial recognition system started late. Under the conditions of insufficient lighting, excessive expression changes, occlusion, high similarity of different individuals, and dynamic recognition, the recognition effect of the facial recognition system cannot reach the ideal expectation. In this paper, the ROI-KNN convolutional neural network face recognition system was studied by using the adaptive quantum genetic algorithm, the improved marker line graph genetic algorithm, and the feature weight value genetic algorithm. The experimental research proved that the recognition effect of the improved ROI-KNN convolutional neural network face recognition system based on the genetic algorithm has been significantly improved.

## Figures and Tables

**Figure 1:** Basic convolution block under ROI-KNN convolutional neural network structure.

**Figure 2:** Architecture of ROI-KNN convolutional neural network.

**Figure 3:** Applications of facial recognition systems.

**Figure 4:** Facial recognition in low-light environments.

**Figure 5:** Facial recognition under different expression changes.

**Figure 6:** Facial recognition under occlusion.

**Figure 7:** Facial recognition under the condition of high degree of face similarity.

**Figure 8:** Facial recognition under dynamic recognition conditions.

**Figure 9:** Facial recognition speed.

**Figure 10:** Facial recognition security.

**Table 1:** Facial recognition under the condition of high degree of face similarity.

	Test group, %	Control group, %
1	69	66
2	71	65
3	79	71
4	80	80
5	85	73

## Data Availability

The data that support the findings of this study are available from the corresponding author upon reasonable request.
